The article "The Correct Localization of Borealin in Midbody during Cytokinesis Depends on IQGAP1" was published in 2020. Journal: Biomed Res Int.

# The Correct Localization of Borealin in Midbody during Cytokinesis Depends on IQGAP1

**DOI:** 10.1155/2020/6231697

**Published:** 2020-06-24

**Authors:** Reziya Wumaier, Abudunaibi Aili, Hexige Saiyin, Pingzhao Zhang, Lihuan Cao, Aikeremujiang Muheremu

**Affiliations:** ^1^State Key Laboratory of Genetic Engineering, Institute of Genetics, School of Life Sciences, Fudan University, Shanghai 200433, China; ^2^Key laboratory of Medical Molecular Virology, Institute of Biomedical Sciences and Institute of Medical Microbiology, Shanghai Medical College, Fudan University, Shanghai 200032, China; ^3^Department of Spine Surgery, Sixth Affiliated Hospital of Xinjiang Medical University, Urumqi, Xinjiang 86830001, China; ^4^Department of Orthopaedics, Peking University Third Hospital, Beijing 86100191, China

## Abstract

Borealin is a key component of chromosomal passenger complex, which is vital in cytokinesis. IQ domain-containing GTPase-activating protein 1 (IQGAP1) also participates in cytokinesis. The correlation between Borealin and IQGAP1 during cytokinesis is not yet clear. Here, we used mass spectrometry and endogenous coimmunoprecipitation experiments to investigate the interaction between IQGAP1 and Borealin. Results of the current study showed that Borealin interacted directly with IQGAP1 both *in vitro* and *in vivo*. Knockdown of IQGAP1 resulted in an abnormal location of Borealin in the midbody. Knocking down Borealin alone, IQGAP1 alone, or Borealin and IQGAP1 at the same time inhibited the completion of cytokinesis and formed multinucleated cells. Our results indicated that IQGAP1 interacts with Borealin during cytokinesis, and the correct localization of Borealin in the midbody during cytokinesis is determined by IQGAP1, and IQGAP1 may play an important role in regulating Borealin function in cytokinesis.

## 1. Introduction

Cytokinesis controls the proper distribution of the replicated cytoplasm and nuclear material in two daughter cells. If this process is abnormal or defective, it will lead to the failure of previous mitotic events and cause cell polyploidy and chromosome instability [1]. In animal cells, cytokinesis usually begins at the anaphase and ends with the complete separation of two daughter cells. After entering the anaphase, the mitotic spindle recompositions to a series of interlaced and antiparallel microtubules, which are called central spindle microtubules. Signals from astral microtubules and central spindle microtubules in centrosome stimulate cells to form a cleavage furrow on the division plane [2]. After the cleavage furrow is formed, the central spindle midzone is reconstructed to form a midbody. The midbody provides an important platform for recruiting and organizing crucial proteins that regulate the detachment of two daughter cells [3]. These midbody proteins can be divided into three subgroups according to their positions: the bulge, the dark zone, and the flanking zone proteins [4].

In the process of cytokinesis, cytoskeleton and many signal proteins need to coordinate to control the dynamic events from the determination of the division plane to the final abscission of two daughter cells. Those proteins include chromosomal passenger complex (CPC), microtubule-associated protein (MAP), and at least three kinesin-like motors, such as KIF4A and KIF20A. Among them, the CPC is mainly composed of Aurora B, INCENP, Borealin, and survivin. At different stages during mitosis, three nonkinase subunits of CPC, Borealin, INCENP, and survivin control the targeting of CPC by directly binding with unique proteins, while Aurora B can phosphorylate different substrates [5]. In the metaphase, CPC is located in the centromere and regulates the arrangement and separation of chromosomes [6]. In the anaphase, CPC activates KIF4A through Aurora B and inhibits microtubule depolymerization enzyme KIF2A and stabilizes the central spindle [7, 8]. During abscission, CPC is located in the midbody [4, 9], and Aurora B kinase phosphorylates the subunit CHMP4C of endosomal sorting complex required for transport- III (ESCRT III) and negatively regulates the process of two daughter cell detachment [10–12]. Interestingly, Borealin is the direct interaction protein between the ESCRT-III subunits Shrb and CHMP4C in Drosophila melanogaster and humans [13, 14]. However, molecular evidence on how CPC regulates the detachment of two daughter cells is still lacking.

Members of the IQ domain-containing GTPase-activating protein (IQGAP) family have four calmodulin binding IQ motifs and a GAP domain for RAS signal transduction [15]. However, those GAP domains do not have a GAP activity due to the lack of arginine finger [16]. In addition to GAP domains, other domains in IQGAPs can also mediate interactions with other proteins [17–19]. IQGAP family proteins exist in many eukaryotes, including *Dictyostelium*, yeast, *Caenorhabditis elegans*, and mammals [20]. The IQGAP homologue Rng2 in *Schizosaccharomyces pombe* and qg1/Cyk1 in *Saccharomyces cerevisiae* is located in the contractile ring of cells and is essential for cytokinesis [21, 22]. IQGAP homologous protein pes-7 in nematode (*C*. *elegans*) also plays important role in cytokinesis [23]. In mammals, three members of the IQGAP family (IQGAP1, IQGAP2, and IQGAP3) have been reported to be essential in cellular activities such as exocytosis, neuronal morphogenesis, cell adhesion, and cell migration [21, 24, 25]. They are also the key regulators in mediating Rho family GTPases and cytoskeleton reorganization. Previous studies have shown that IQGAP1 stabilizes the active forms of RAC1 and CD42 [26, 27] IQGAP family is closely linked to small GTPase network; IQGAP1 interacts with several small GTPases and their network proteins [28]. IQGAP1 seems to accumulate at the contractile ring and activate RhoA in the equatorial cortex [29]. The expression of IQGAP1 mutant in HeLa cells resulted in the formation of multinucleated cells [30]. In the current study, we hypothesized that IQGAP1 interacts with Borealin during cytokinesis and found that IQGAP1 colocalized with Borealin in the midbody, and the correct location of Borealin in the midbody depends on the interaction with IQGAP1.

## 2. Materials and Methods

### 2.1. Cell Culture

HeLa cells transfected with pCIN4-Flag-HA-Borealin and HeLa cells transfected with the control vector were cultured in DMEM containing 10% fetal bovine serum (FBS) at 37°C and 5% CO_2_.

### 2.2. Plasmid Constructs and siRNA Fragments

Full-length Borealin cDNA (CDCA8) was kindly provided by Dr. Ulrike Gruneberg (University of Oxford) and cloned into pCIN4-Flag–HA and pCMV-HA/Myc/His vectors. Human EGFP-C1-IQGAP1 was provided by David B Sacks from the National Institutes of Health and then cloned into pGex-4T-1vector. The siRNA target sequences in the sense orientation were as follows:

IQGAP1-1: 5′- GGAUGAAGCCGCAUUACAdTdT-3′;

IQGAP1-2: 5′- GCUGAAAUUCAAGGCAAUdTdT-3′;

Borealin-1: 5′- CGGAGAGAGCCUGCGAUUAUUdTdT-3′;

Borealin-2: 5′-CCUGGAUAUCACCGAAAUAAAdTdT-3′;

siControl: 5′-CGUACGCGGAAUACUUCGAdTdT-3′.

### 2.3. Cell Transfections

Cells were seeded at 40–50% confluence. For DNA transfections, cells were transfected with 0.3 *μ*g and 0.6 *μ*g of the indicated plasmid DNA per well, using Lipofectamine 2000 (Invitrogen). For siRNA analyses, cells were transfected with 0.05 *μ*M of siRNA oligos using Lipofectamine RNAiMAX (Invitrogen).

### 2.4. Immunoprecipitation and Western Blotting

HeLa cells were washed with PBS, then lysed in ice-cold BC100 lysis buffer for 20 min on ice. After centrifugation at 13,000 rpm for 20 min at 4°C, the supernatant was incubated with antibody at 4°C 12 h, washed six times with BC100 buffer, and then incubated with protein A/G beads for 4 h at 4°C. After six washes with BC100 buffer, cell lysates or immunoprecipitates were subjected to SDS-PAGE and transferred to nitrocellulose membranes. The membranes were first blocked with Tris-buffered saline (TBS, pH 7.4) containing 0.1% Tween-20 and 4% nonfat milk, and then incubated with primary antibody for at 4°C 12 h, and lastly incubated with secondary antibody for 3 h at 4°C. And then, ECL chemiluminescence system (Santa Cruz) was used for detecting proteins.

### 2.5. Antibodies

Commercially available antibodies were as follows: anti-Borealin (Santa Cruz Biotechnology) 10 *μ*g/mL for western blot and immunofluorescence 5 *μ*g/mL, anti-IQGAP1 (Santa Cruz Biotechnology) 1 *μ*g/mL for western blot and immunofluorescence 2 *μ*g/mL, anti-Aurora B (BD Biosciences) 6 *μ*g/mL for immunofluorescence, anti-*α*-tubulin (Abcam) 5 *μ*g/mL for immunofluorescence, anti-*β*-tubulin (Abcam) 5 *μ*g/mL for immunofluorescence, and anti-*β*-actin (AC-74, Sigma) 0.1 *μ*g/mL for western blot.

### 2.6. Protein Complex Purification

HeLa cells were transfected with pCIN4-Flag-HA-Borealin constructs and selected for 3 weeks in 1.5 mg/mL G418. The tagged Borealin protein levels were detected by western blot. The stable cell lines that express Flag-HA-Borealin were chosen to expand. For protein complex purification, the HeLa/Borealin cells were lysed in BC100 buffer (20 mM Tris-Cl, pH 7.5, 20% glycerol, 100 mM NaCl, and 0.2 mM EDTA) containing 0.1% Triton X-100 and protease inhibitor on ice for 4 h. After centrifugation for 40 min with 12500 rpm at 4°C, the supernatant of the cell lysates was immunoprecipitated by anti-Flag antibody-conjugated M2 agarose (Sigma). After washing three times with the BC100 buffer to remove the unbounded protein, immunoprecipitated by anti-HA antibody-conjugated M2 agarose (Sigma), the bound polypeptides were eluted with peptide and resolved by SDS-PAGE for Coomassie Blue staining. Gel lanes (strips) were subjected to mass spectrometric sequencing.

### 2.7. Purification of Recombinant Protein

The recombinant GST-IQGAP or His- Borealin was expressed in Escherichia coli strain BL21-CodonPlus (DE3)-RIL with 0.5 mM IPTG (isopropyl- *β*-D-thiogalactopyranoside) at 23°C after 12-hour and 16-hour induction, respectively. Cells were collected and lysed, and the GST recombinant protein and His recombinant protein were purificated as previously described [31].

### 2.8. GST Pull-Down Assay

GST-IQGAP protein was immobilized on Glutathione Sepharose 4B (Amersham Biosciences). After washing with pull-down buffer (25 mM Tris-HCl, pH 7.5, 10% glycerol, 0.1% NP-40,150 mM NaCl, 1 mM EDTA, 1 *μ*g/mL leupeptin, and 1 mM DTT), the beads were incubated with recombinant His-borealin for 3 h at 4°C. The beads were then washed six times with a binding buffer. The bound proteins were then resuspended in sample buffer for SDS-PAGE and western blot analysis.

### 2.9. Immunofluorescence and Confocal Microscopy

For immunofluorescence tests, cells were plated on chamber slides and fixed with 4% paraformaldehyde for 25 min at 23°C. To examine the immunofluorescence of protein at each mitotic stage, cells were synchronized by double-thymidine block and release to fresh media. A staging system was used to identify the different phases of mitosis based on the DNA and extent of chromosome alignment and separation, which was described in our previous publication [32]. For example, when after double-thymidine block cells were released by fresh media, they entered the M-phase, and 8 hours after releasing the cells into fresh media, they reached cytokinesis [32]. After fixation, cells were permeabilized with 0.2% Triton for 5 min, blocked with 5% goat serum in PBS. The cells were incubated with primary antibody solutions at 4°C overnight. Slides were washed, incubated with fluorescence-tagged secondary antibodies (Alexa Fluor 488, 568, Molecular Probes, Invitrogen), and counterstained with DAPI (Vector Labs) for 1 h at 4°C. Images were acquired using a Zeiss LSM710 confocal microscope equipped with a 60x objective. Fluorescence from multiple planes throughout the cells were collected to create a stack of two-dimensional (2D) images (*z*-stack); each plane showing fluorophore localization on the *x* and *y* planes; those planes were computationally reconstructed to form the 3D image of the cells, which were then projected as a 2D view on a computer screen [33]. For time-lapse imaging, Zeiss TRIF fluorescent live cell imaging microscope equipped with a 20x objective was used. Images of proteins of interest were acquired using identical imaging settings. Image processing and figures were made using PhotoShop CS (Adobe).

## 3. Results

### 3.1. Borealin Interacts with IQGAP1 Both In Vitro and In Vivo

The HeLa monoclonal cell line was constructed with stably expressing Flag-HA-tagged Borealin protein, after treatment with double-thymidine block (DTB); cells whose division process synchronized to cytokinesis were collected. After tandem affinity purification (Figure 1(a)), the complex formed by Borealin protein was analyzed by mass spectrometry. We identified IQGAP1 as one of the Borealin-interacting proteins, and its score was comparable to or higher than the other members of CPC, survivin, INCENP, and Aurora B (Table 1).

IQGAP1 is an important component in a small GTPase network and plays a key role in cytokinesis. To find the relationship between IQGAP1 and Borealin in cytokinesis, we first investigated whether the interaction between IQGAP1 and Borealin is direct. Recombinant GST-IQGAP1 protein and His-Borealin protein were expressed and purified, respectively, in bacteria. As shown in Figure 1(b) and 1(c), GST-IQGAP1, but not single GST, binds to His-Borealin in the pulled-down complex, indicating that IQGAP1 and Borealin interact physically. Then, we used endogenous immunoprecipitation to detect whether IQGAP1 interacted with Borealin in HeLa cells. As shown in Figure 1(d), Borealin was detected in anti-IQGAP1 immunoprecipitates by western blotting, and IQGAP1 was also detected in anti-Borealin immunoprecipitates. Therefore, our data demonstrate that Borealin directly interacts with IQGAP1 both in vitro and in vivo.

### 3.2. IQGAP1 Colocalized with Borealin and Aurora B in the Midbody

We then observed the subcellular localization of Borealin and IQGAP1 at different stages of HeLa cell division by two-dimensional immunofluorescence assay analysis. We found that Borealin changed its position during cell cycle progression. In the interphase, Borealin was found in the nucleus; in the prophase, Borealin was enriched in the centromere; in the metaphase, it is mainly located in the equator and centromere; in the anaphase, it was mainly located in the central spindle area and cleavage furrow (Figure 2(a)). Borealin was located in the arm of the midbody during the formation of the intercellular bridge between the two daughter cells (Figure 2(a)). As for IQGAP1 protein, we found that it was enriched in cell membrane during the interphase, prophase, and metaphase, and it was enriched in the cleavage furrow at the anaphase and telophase. IQGAP1 was also enriched in the midbody during the formation of bridges between two daughter cells (Figure 2(b)).

In view of their coherent enrichment in the cleavage furrow and cytokinesis midbody at later stages of cell division, analyzing the three-dimensional reconstruction images of cells that were projected to two dimensional plane, we noticed the colocalization of Borealin and IQGAP1 at different stages of cell cycle, and immunofluorescence tests indicated that Borealin and IQGAP1 were colocated in the cleavage furrow (Figure 3(a)) and midbody (Figure 3(a)).

We also observed that the colocalization of other CPC members Aurora B and IQGAP1 (Figure 3(b)), Borealin and Aurora B, Borealin and IQGAP1, and IQGAP1 and Aurora B were colocalized in the midbody. Interestingly, Aurora B, Borealin, and IQGAP1 were all located in the flanking region of the midbody. Meanwhile, IQGAP1 was also located more outside of the flank region, not close to the dark area, compared with Aurora B and Borealin. These results of colocalization in the midbody suggest that IQGAP1 with CPC complex may functionally regulate each other during cytokinesis.

### 3.3. Location of Borealin in Midbody Depends on IQGAP1

In order to study the functional significance of the interaction between Borealin and IQGAP1, we first analyzed the location of IQGAP1 after Borealin was knocked down. We found that Borealin knockdown resulted in the failure of cell division from the metaphase to anaphase and the inability of the duplicated sister chromatids to separate, leading to considerable distortions in cell structure (Figure 4). We believe that this is related to the dynamic localization of CPC complexes in the process of cell division and their multiple functions. Therefore, we could not reach a conclusion on the distribution of IQGAP1 during cytokinesis after Borealin was depleted.

When analyzing the location of Borealin after the knockdown of the IQGAP1 protein, we found that the localization of Borealin was disturbed in the midbody. Borealin was located in only half of the flank region close to the dark area, but not in the lateral region of the flank, which was the position of IQGAP1 in the midbody (Figure 5). In the control cells, Borealin was located in the entire flanking region of the midbody. Therefore, it is safe to assume that the correct location of Borealin in the midbody depends on the IQGAP1 protein.

### 3.4. IQGAP1 May Play an Important Role in Regulating Borealin Function in Cytokinesis

Finally, we studied the functions of Borealin and IQGAP1 in cytokinesis. When Borealin or/and IQGAP1 was knocked down in HeLa cells, cytokinesis could not be completed, leading to the formation of multinucleated cells. When we knocked down Borealin using two different siRNA-targeting sequences, it resulted in a 33% increase in the proportion of polynuclear cells. In the meanwhile, knockdown of IQGAP1 in HeLa cells resulted in a 12% increase in the percentage of polynuclear cells. When IQGAP1 and Borealin were knocked down together, the percentage of polynuclear cells was 30-35%, similar to that of Borealin knock down (Figure 6). Borealin depletion results in the failure of entering cytokinesis, and its location during cytokinesis depends on IQGAP1, so these data suggest that IQGAP1 may play an important role in regulating Borealin function in cytokinesis.

## 4. Discussion

Proteomics and cell biology studies have shown that more than 100 proteins are located in the convex, dark, and flanking regions of the midbody. The midbody is vital as a platform for these proteins to regulate the final detachment of two daughter cells [3, 23]. It has been known that the CHMP4C subunit of the endosomal sorting complex ESCRT-III can be assembled into helical filaments only when the CPC accumulated in the flanking region of the midbody is removed. This CPC-mediated ESCRT-III regulation is thought to be a cell division checkpoint to prevent the midbody from splitting and detaching when DNA is present, thus avoiding the formation of genetically abnormal daughter cells. However, molecular evidence lacks on how CPC regulates the detachment of two daughter cells.

Borealin, a member of CPC complex, interacts with subunits CHMP4A, CHMP4B, and CHMP4C of ESCRT-III. Therefore, we constructed a Flag-HA double-tagged and Borealin overexpressing cell line, collected cells whose division process synchronized to the cytokinesis stage, and investigated Borealin-interacting proteins in the cytokinesis process to find the key regulator proteins. We identified IQGAP1 as a Borealin-interacting protein during cytokinesis and found that IQGAP1 colocalized with Borealin in the midbody, and the location of Borealin in the midbody depended on its interaction with IQGAP1.

Aurora B, a member of the CPC complex, phosphorylated CHMP4C during cytokinesis, and high Aurora B activity delays the final detachment [10, 11, 34] Another study revealed that the interaction between Aurora B function and citron kinase have a synergic effect on cytokinesis [31] It was also found that ANCHR (abscission/no cut checkpoint regulator; ZFYVE19) is an interacting protein of Aurora B and a key regulatory factor for detaching from the checkpoint [35]. In the current study, we also found that Aurora B was colocalized with Borealin-interacting protein IQGAP1, and location of Aurora B in midbody was disrupted when IQGAP1 was knocked down (data not shown). Depletion of IQGAP1 may impare the stability of CPC complex members in the midbody.

Although other members of IQGAP family and IQGAP1 are generally considered to be related to cytokinesis [29, 30], the detailed function of other IQGAPs in cytokinesis is not yet clear. Adachi et al. [36] reported that IQGAP3, rather than IQGAP1, is mainly involved in the formation of contractile rings during cytokinesis. Another study proposed that IQGAP1 participated in reassembling nuclear pore complexes during cytokinesis [37]. Our data indicated that IQGAP1 is located in the midbody, while Aurora B and Borealin were all located in the flanking region. This colocalization at the midbody is presented with CPC components occupying the central region and IQGAP1 decorating halfway down the midbody arms. In our experiments, knocking down Borealin would lead to the failure of transition from the metaphase to anaphase, causing the formation of polynuclear cells. Meanwhile, knocking down IQGAP1 affected the normal location of Borealin in the midbody, then caused the failure of cytokinesis and formed polynuclear cells. While Borealin is the main component of cellular division, IQGAP1 affects cell division by controlling the location of Borealin during the final abscission of two daughter cells. We believe that is the reason why after simultaneously knocking down both Borealin and IQGAP1, there was no further increase of polynuclear cells than knocking down Borealin alone.

Our results provide preliminary evidence of functional links between CPC complexes and IQGAP1 during cytokinesis. Results of the current study can be further translated to find drug targets for tumorigenesis and innate immunity [38–40]. Meanwhile, more cell lines are required in the future to further investigate this correlation, and further research is needed to study the role of IQGAP in stabilizing the CPC and the mechanism of how CPC and IQGAP1 play coordinated role during the completion of cytokinesis.

## 5. Conclusion

Our results indicate that IQGAP1 interacts with Borealin during cytokinesis and plays key role in cell division, and the correct localization of Borealin in the midbody is determined by IQGAP1.

## Figures and Tables

**Figure 1:** IQGAP1 interacts with Borealin both *in vivo* and *in vitro.* (a). Tandem affinity purification of Borealin-containing protein complexes was conducted using HeLa cells stably expressing Flag-HA- (FH-) Borealin and the control group with an empty vector. The protein complex was separated by SDS-PAGE and visualized by Coomassie Blue (CB) staining. The proteins and the number of peptides identified by mass spectrometry are shown in Table 1. (b) Purified His-Borealin from bacteria was incubated with GST-IQGAP or GST that was prebound to glutathione agarose beads. Half of the binding proteins from these beads were separated by SDS-PAGE and visualized by CB, and half were detected by western blotting with anti-His antibody. (c) Purified His-Borealin was separated by SDS-PAGE and visualized by CB. (d) The endogenous Borealin was immunoprecipitated by anti-Borealin antibody, and the immunoprecipitates were detected by western blotting with the indicated antibodies. Endogenous IQGAP1 was immunoprecipitated by anti-IQGAP1 antibody, and the immunoprecipitates were detected by western blotting with the indicated antibodies. Three independent biological replicates were performed in the purification of recombinant protein and immunoprecipitation experiments.

**Figure 2:** Dynamic localization of Borealin and IQGAP1 during mitosis in HeLa cells. (a) HeLa cells synchronized by double-thymidine treatment were fixed and stained with Borealin antibody (green), alpha-tubulin antibody (red), and DAPI (blue) or (b) IQGAP1 antibody (green) and alpha-tubulin antibody (red), and DAPI (blue). Three independent biological replicates were performed.

**Figure 3:** IQGAP1 colocalized with Borealin and Aurora B at the midbody.(a) HeLa cells synchronized by double-thymidine treatment were fixed and stained with IQGAP1 antibody (green), Borealin antibody (red), and DAPI (blue). (b) Colocalization of IQGAP1, Borealin, and Aurora B at the midbody. (A) HeLa cells synchronized by double-thymidine treatment were fixed and stained with Borealin antibody (green), Aurora B antibody (red), and DAPI (blue); or (B) IQGAP1 antibody (green), Borealin antibody (red), and DAPI (blue); or (D) IQGAP1 antibody (green), Aurora B antibody (red), and DAPI (blue). Bar = 10 *μ*m.

**Figure 4:** Borealin depletion distorted the cell's architecture. (a). HeLa cells were treated with siRNAs against Borealin or control. After 48 h, cell lysates were detected by western blotting with the indicated antibodies. (b). HeLa cells were treated with siRNAs against Borealin or control. After 48 h, cells were fixed and stained with IQGAP antibody (green), alpha-tubulin antibody (red), and DAPI (blue). Bar = 10 *μ*m. (c). The HeLa cell line with stably expressing mCherry-H2B was treated with siRNAs against Borealin or control. After 48 h, time-lapse imaging was used to observe the process of cell division. (d). Statistic diagram of the time required for cells from nuclear envelope breakdown (NEBD) to the anaphase.

**Figure 5:** Localization of Borealin in the midbody depends on IQGAP1. (a). HeLa cells were treated with siRNAs directed against IQGAP1 or control. After 48 h, cell lysates were detected by western blotting with the indicated antibodies. (b). HeLa cells were treated with siRNAs direct against IQGAP1 or control. After 48 h, cells were fixed and stained with Borealin antibody (green), alpha-tubulin antibody (red), and DAPI (blue). Bar = 10 *μ*m. The graph below shows the overlap of fluorescence intensity peaks along profile localization of Borealin on midbody in the merged micrograph. (c) The percentage of Borealin midbody location disturbed in IQGAP1-depleted cells and in control cells. A minimum of 150 cells were counted per sample in three independent experiments. Error bars represent ±S.E.

**Figure 6:** IQGAP1 and Borealin codepletion inhibits cytokinesis completion. (a) HeLa cells were treated with siRNAs directed against Borealin and IQGAP1 together or control. After 48 h, cell lysates were detected by western blotting with the indicated antibodies. (b) RNAi-mediated silencing of Borealin and IQGAP1 together induced multinucleation in HeLa cells. After 48 h, cells were fixed and stained with tubulin antibody (green) and DAPI (blue). (c) IQGAP1 and Borealin codepletion inhibits cytokinesis completion. HeLa cells were individually treated with siRNAs against *Borealin* alone, *IQGAP1* alone, or *CDCA8* and *IQGAP1* together, and were fixed after 72 h. At least 400 cells were counted every time from three independent experiments. Error bars indicate S.D. *Error bars* represent ±S.E. ^∗∗∗^*p* < 0.001; *n.s.*, not statistically significant.

**Table 1:** Summary of mass spectrometry results from the affinity purification of Flag-HA-tagged Borealin. Several proteins identified from the affinity purifications are listed along with their relative Mascot score and number of peptides.

Proteins	Score	Peptides
Borealin	4462	19
GRP78	4105	35
IQGAP1	3006	27
ATBP	2093	18
KIF11	2091	26
BIRC5	522	5
INCENP	371	8
AURKB	85	2

## Data Availability

All data generated or analyzed during this study are included in this published article.
